The article "Sparse Dictionary-Based Magnetic Resonance Superresolution Imaging with Joint Loss Function Learning" was published in 2022. Journal: J Healthc Eng.

# Sparse Dictionary-Based Magnetic Resonance Superresolution Imaging with Joint Loss Function Learning

**DOI:** 10.1155/2022/2206454

**Published:** 2022-08-29

**Authors:** Huanyu Liu, Xiaodong Liu, Jinyu Wu, Lu Li, Mingmei Shao, Yanyan Liu

**Affiliations:** ^1^Information Countermeasure Technique Institute, School of Computer Science and Technology, Harbin Institute of Technology, Harbin 150080, China; ^2^Department of Automatic Test and Control, School of Electronics and Information Engineering, Harbin Institute of Technology, Harbin 150080, China; ^3^Harbin the First Hospital, Harbin 150010, China; ^4^Defence Industry Secrecy Examination and Certification Center, Beijing 100001, China; ^5^Science and Technology on Electro-Optical Information Security Control Laboratory, Tianjin, China

## Abstract

Magnetic resonance image has important application value in disease diagnosis. Due to the particularity of its imaging mechanism, the resolution of hardware imaging needs to be improved by increasing radiation intensity and radiation time. Excess radiation can cause the body to overheat and, in severe cases, inactivate the protein. This problem is expected to be solved by the image superresolution method based on joint dictionary learning, which has good superresolution performance. In the process of dictionary learning, the loss function will directly affect the dictionary performance. The general method only uses the cascade error as the optimization function in dictionary training, and the method does not consider the individual reconstruction error of high- and low-resolution image dictionary. In order to solve the above problem, In this paper, the loss function of dictionary learning is optimized. While ensuring that the coefficients are sufficiently sparse, the high- and low-resolution dictionaries are trained separately to reduce the error generated by the joint high- and low-resolution dictionary block pair and increase the high-resolution reconstruction error. Experiments on neck and ankle MR images show that the proposed algorithm has better superresolution reconstruction performance on ×2 and ×4 compared with bicubic interpolation, nearest neighbor, and original dictionary learning algorithms.

## 1. Introduction

Magnetic resonance (MR) imaging is widely used in medical application and plays an increasingly important role in the diagnosis of various diseases. When applying MR imaging, a RF pulse of a specific frequency is applied to the human body in a static magnetic field, exciting hydrogen protons in the human body; thus the magnetic resonance phenomenon occurs [1, 2]. After stopping the pulses, the proton generates MR signals during relaxation. MR images are generated by MR signal reception, spatial encoding, and image reconstruction [2, 3] and have been used in imaging diagnosis of various systems throughout human body, including cranium, brain, spinal cord, cardiovascular, articular cartilage, soft tissue, pelvic, etc. [4, 5].

In practical applications, images of high resolution usually provide more details of the image, which can be very useful for subsequent image processing. Although hardware with better performance can be used to improve image resolution, many researchers prefer to adopt image superresolution reconstruction technology due to cost and technical limitations. Superresolution reconstruction technology refers to the reconstruction of a corresponding high-resolution image from one or more low-resolution images, which is mainly based on methods including interpolation, reconstruction, and learning [6–8]. According to [9–11], the image interpolation method is to estimate the unknown pixels among the known pixels according to the law of the pixels in a limited area. Traditional interpolation model does not consider the image degradation model and mainly includes nearest neighbor interpolation, bilinear interpolation, and bicubic interpolation. The image superresolution method based on interpolation is simple and efficient and can meet the requirements of real-time application. However, such methods take into account the local structure characteristics of the low-resolution image itself, resulting in distortion in areas with rich texture. Especially in the case of large magnification, the reconstructed image will have serious degradation and blurring phenomenon, and the visual quality of the image will be greatly reduced. Essentially, the interpolation method does not add more information to the image. The method based on reconstruction assumes that the low-resolution image can well predict the original high-resolution image. This method mainly takes the prior knowledge of the image as the constraint to estimate high-resolution image, including methods such as Iterative Backprojection (IBP), Maximum Posterior Probability, Projection Onto Convex Sets (POCS), etc. [12–14]. Most of these methods use the prior knowledge of images such as edge characteristics, nonnegativity of pixels, and local smoothing characteristics. We use the prior knowledge to construct constraint conditions and then solve the optimization problem through iterative algorithm. This results in the insufficient use of the prior information of the image, and when the amplification factor is large, the reconstructed image is often too smooth [15, 16]. According to the previous work [17, 18], image prior information that is more effective has been widely used in recent years, such as self-similarity, sparsity, etc. The computational complexity of the algorithm was increased.

Learning-based methods include methods based on manifold learning, dictionary learning, and deep learning. Essentially, the learning-based method is to learn the mapping relationship between low-resolution images and high-resolution images, so as to increase the information of low-resolution images. The method based on Manifold Learning assumes that high-resolution image blocks and low-resolution image blocks are used to form two manifolds with similar local geometric features in the feature space. The feature vector of an image block is extracted by local geometric features and can be reconstructed from adjacent data points in feature space, and the local compatibility and smoothness of the target high-resolution image are guaranteed by the overlap between the image blocks according to Manifold Learning [19]. Dictionary Learning is based on sparse representation theory, and its purpose is to find a code with complete basis set composition (that is, to extend to the whole image space). We find the expression coefficients that are independent from each other as far as possible in the image, that is, to ensure that the extracted basis is the essential feature of the signal. We must consider two constraints when using dictionary learning for superresolution image reconstruction: firstly, reconstruction constraint, that is, the reconstructed image is required to be consistent with the input image after passing the degradation model; secondly, sparse prior constraint, that is, high-resolution image blocks can be sparsely represented using high-resolution dictionaries, and this sparse representation can be recovered from the corresponding low-resolution dictionary sparse representation of low-resolution image blocks. In the reconstruction constraint, we obtain the low-resolution image through the high-resolution image obtained after fuzzy and downsampling operation. In the joint learning of high- and low-resolution dictionaries, only the cascading error is generally considered, not the reconstruction error of high-resolution image [20]. The joint dictionary learning superresolution method is also applied to MR image. Andrea et al. [21] put forward such MR image superresolution reconstruction based on sparse representation framework, and MR images shall be carried out in accordance with the regional segmentation of gray matter, white matter, and cerebrospinal fluid; adjacent areas from different parts of the image block are chosen as the training set, to consider the whole image multiscale edge analysis and dimension reduction scheme, significantly improving the calculation speed and accuracy. Zhang et al. [22] jointly used sparse prior, nonlocal similarity, and sparse derivative prior to MR image superresolution. Multiscale first and second derivatives are used to estimate high-frequency information, and sparse derivative priority-based postprocessing is used to suppress the fuzzy effect in MR images. Kaur and Sao [23] proposed a constraint method for sharpening the gradient distribution of superresolution MR images within the superresolution framework based on sparse representation. By establishing a piecewise linear relationship between the gradient distribution of low-resolution images amplified by bicubic interpolation and corresponding low-resolution images, the gradient distribution of upsampled low-resolution images is improved, and the superresolution of MR images is realized. Huang et al. [24] proposed an exotic image alignment term in order to combine unpaired data from different image resolutions/modes. Local image neighborhoods can be naturally preserved by operating on the whole image domain (as opposed to image blocks) and using joint convolution sparse coding. Paired images are enhanced by unpaired data and additional maximum mean difference terms during joint learning, which minimizes differences between their feature distributions.

With the popularity of deep learning, it has gradually expanded to the field of image superresolution. At present, the commonly used deep superresolution networks mainly include three categories: Feedforward Deep Network, Feedback Deep Network, and Generative Adversarial Network [25]. For example, feedforward depth network DBPN [26] provides an error feedback and interdependence method. This method uses image degradation and high resolution and uses the characteristics of phase to improve the performance of SR. The feedback depth network RDN [27] uses dense connected convolution layer to extract rich local features. SRFBN [28] implements this feedback method with hidden state in constrained RNN. As the feedback depth network, EDSR [29] applies the batch normalization (BN) operation. The generative countermeasure network SRGAN [30] takes the residual network as the main network of feature extraction and adds the perceptual loss function. Reference [31] proposed an image superresolution reconstruction method using attention mechanism with feature map to facilitate reconstruction from original low-resolution images to multiscale superresolution images. All these representative networks perform well on natural images SR. At present, the researcher presented some deep learning methods to the superresolution processing of MR images [32]. Oktay et al. [33] proposed a new image superresolution method based on residual convolution neural network model. Hyun et al. [34] proposed a deep convolution network based on *K*-space data mapping on the basis of U-NET network to map undersampled data in *K*-space to MR images. In order to ensure the invariance of original *K*-space data, a data consistency prior was introduced to make reconstructed MR images have better perceptual effects. Xue et al. [35] proposed a progressive subband residual learning superresolution network (PSR-SRN), which consists of two parallel progressive learning flows, one of which flows through the subband residual learning unit to learn the missing high-frequency residual, and the other flow focuses on the reconstruction of refined MR images. The two learning streams complement each other and learn complex mappings between high- and low-resolution MR images. Zhang et al. [36] proposed a new hybrid network that improves the quality of MR images by increasing the width of the network. The hybrid block combines multipath structure and mutation dense block to extract rich features from low-resolution images. Tan et al. [37] combined the meta-learning technology of [38] with GAN network to achieve superresolution of MR images with arbitrary scale and high fidelity. Reference [39] applies DENSENET to the superresolution of brain MRI images. 3D CNN architecture provides more texture details. Then, the performance of deep learning superresolution network is directly affected by the amount of data. Since it is difficult to obtain large amount of MR image data, we prefer to adopt the joint dictionary learning framework for MR image superresolution.

For this paper, the main contributions are as follows: (1) We propose a superresolution architecture based on joint dictionary learning suitable for a small number of MR images. (2) We propose an error loss function based on reconstruction quality constraints, adopt the independent calculation of the reconstruction error of the high- and low-resolution dictionaries, consider the individual reconstruction errors of the high- and low-resolution dictionaries, abandon the traditional cascade calculation method, effectively reduce the reconstruction error, and solve the traditional reconstruction error. The dictionary joint cascade training does not consider the problem of individual reconstruction errors of high- and low-resolution dictionaries. (3) Experiments prove that our proposed method can achieve state-of-the-art performance, even if there is only a less image data.

## 2. The Architecture of MR Image Superresolution Algorithm

### 2.1. The Framework of Superresolution Algorithm

Under the framework of the MR superresolution reconstruction based on joint dictionary learning, we apply the pretrained high-resolution dictionary and low-resolution dictionary. We create the low-resolution image training sets with the image degradation of the corresponding image in the high-resolution image training set. The high and low part of the dictionary block of the trained joint dictionary are one-to-one, by calculating the sparse representation coefficient of the low-resolution input image or the image feature block with respect to the low-resolution dictionary, to restore the corresponding high-resolution image blocks and reconstruct images. In order to ensure the effectiveness of the block-to-block connection of the reconstructed image, the reconstructed image blocks need to overlap to meet the reconstruction constraints between the blocks, so that the reconstructed image block is consistent with the original image block in the reconstruction area. On the other hand, we train the joint dictionary with the probability model. In order to ensure that the image blocks have the same sparse representation of the high-resolution dictionary and the low-resolution dictionary, the image blocks are concatenated and normalized, and then the input dictionary training algorithm is performed at the same time. The image superresolution algorithm is to represent the image block of the input image block. We choose the dictionary element that best represents the characteristics of the input image block from the dictionary. The number of dictionary elements is variable, and the high-resolution image reconstructed by searching for high-resolution image blocks based on this sparse representation has clearer texture and edge and better robustness. The MR superresolution reconstruction framework based on joint dictionary learning is shown in Figure 1.

In the superresolution image reconstruction, the sparse representation of the dictionary of the input image block needs to be calculated. The dictionary uses the selected image to obtain the information (such as edge and texture) that best represents the essential features of the image in the image training block through the dictionary training algorithm and stores it in the form of image block vector. The task of superresolution is to enhance the resolution of image and make the image appear locally compatible and natural, with obvious edge texture information. Since the human eye is most sensitive to the high-frequency details in the image, the task of superresolution is to increase the high-frequency details in the enlarged image that did not exist before. The process of using the existing information of the low-resolution image to predict the high-frequency details of the enlarged image needs the basis of prediction, and the basis is the dictionary. The process of dictionary training is to preprocess a certain kind of image set, extract the details (such as edges and textures) of high-resolution images, sample image blocks, and obtain the training data set through the dictionary training. The dictionary obtained through training is redundant dictionary, in which the number of bases is far greater than the dimension of each basis, and each atom represents some detail information of the image.

The dictionary can reduce the size of the data set, thus greatly reducing the calculation amount of the image superresolution algorithm. If the original image features are directly used to carry out the superresolution algorithm, the computational efficiency will be low due to the huge amount of data. In addition, the dictionary is trained to ensure that all the features of image blocks exist in the dictionary, and the dictionary is redundant; that is, different image blocks to be represented have several representations. Searching the most sparse representation according to the dictionary is beneficial to high-resolution image reconstruction.

### 2.2. Sparse Representation and Reconstruction

#### 2.2.1. Sparse Representation

For image data, if *I*(*x*, *y*) is an image signal, then it can be expressed as a linear superposition of the basis function *ϕ*_*i*_(*x*, *y*).

(1) $$\begin{array}{c} I\left(x,y\right)=\underset{i}{\sum }\alpha_{i}\phi_{i}\left(x,y\right). \end{array}$$

*α*_*i*_ is the sparsity coefficient corresponding to each basis function. The image coding depends on the basis function, while the sparsity coefficient *α*_*i*_ changes with different images. The purpose of sparse representation is to find a complete coding of the base set (that is, to extend to the entire image space) and to find the expression coefficients which are as independent to each other as possible in the image, that is, to ensure that the extracted basis functions are the essential features of the image.

The meaning of signal sparsity is that the original signal is decomposed and represented sparsely in a specific overcomplete signal feature space (sparse representation), and the signal, which is represented by the selected feature component through linear combination, meets the requirement of proximity with the original signal on the condition that their error (represented by mean-square deviation) is within the prescribed margin of error. Under this circumstance, the number of features selected from the feature space represents the sparsity.  Figure 2 is the sparse structure representation of MR images, in which the image block array is part of the “basis function” obtained after feature extraction of randomly selected image blocks from MR images. A test image block is selected and sparse decomposition is performed according to (1). Three feature blocks are selected from the test image block; i.e., the sparsity is 3. The image block gradient feature is selected here because the combination of gradients in different directions can describe the whole image.

#### 2.2.2. Image Reconstruction

The reconstruction process of joint dictionary image is based on the input single low-resolution image, using the pretrained joint dictionary to obtain the sparse representation system, so as to obtain the high-resolution reconstructed image of the corresponding scene. It is assumed that *D* ∈ *R*^*n*×*K*^(*K*〉*n*) is an overcomplete dictionary containing *K* atoms, and the input image signal *x* ∈ *R*^*n*^ can be represented by a linear combination of dictionary *D*, and the sparse representation meets the sparse condition.

(2) $$\begin{array}{c} x=D\alpha ,\overset{K}{\underset{i=1}{\sum }}{\left|\alpha_{i}\right|}^{0}\ll K. \end{array}$$

Assume that *L* is a mapping matrix, representing the degradation process of the image; then the degradation process of the image can be expressed by the following formula, in which *x* is the high-resolution image, and *y* is the corresponding low-resolution image. Equations (2) and (3) are underdetermined matrix, based on compressed sensing theory; in (3) the solution of *α*_0_ is unique under weak condition. And if the dictionary meets the near isometric condition, for different kinds of degradation matrices, the sparse representation coefficients of any linear combination of high-resolution image *x* can be perfectly reconstructed from low-resolution images.

(3) $$\begin{array}{c} y=Lx=LD\alpha ,\;L\in R^{k\times n}\left(k<n\right). \end{array}$$

When reconstructing high-resolution image *x* of the corresponding scene of a single low-resolution image *y*, two constraints need to be considered: (1) reconstruction constraints, that is, the reconstructed image *x* is required to be consistent with the input image *y* after *x* passing through the degradation model; (2) sparse prior constraints, that is, a high-resolution image block can be sparsely represented by a high-resolution dictionary, and the sparse representation can be restored from a low-resolution dictionary sparse representation corresponding to a low-resolution image block. In the process of reconstructing a superresolution image, firstly, a sparse prior is used to calculate the sparse representation of the local image block under the condition of compatibility between adjacent blocks, and then the sparse representation is used to reconstruct the entire image under the condition of satisfying the reconstruction constraints. Essentially, the local model of sparse prior here is used to find the high-frequency detail information of the local image block, and the global model of reconstruction constraint is used to remove any possible artificial errors to make the image more continuous and natural.

When obtaining the sparse representation of the input image block, the image needs to be preprocessed so that the low-resolution image block to be sparsely represented represents texture information, and then the sparse representation of the texture information of the low-resolution image block concerning dictionary *D*_*l*_ is solved as formula (4):

(4) $$\begin{array}{c} \min{\left\|\alpha \right\|}_{0},\\ \text{s.t.}{\left\|FD_{l}\alpha -Fy\right\|}_{2}^{2}\leq \varepsilon . \end{array}$$

In formula (4), ‖.‖_0_ is the 0 norm, which represents the sparsity of the sparsity coefficient *α*, ‖.‖_2_^2^ is the square of the 2 norm, which represents the sparse approximation error of the low-resolution local image block, *F* is the feature operator for extracting the image texture detail information, and *ε* is a small constant. The optimization of formula (4) is an NP problem. When the main sparseness is sufficiently sparse, formula (4) can be effectively restored using formula (5).

(5) $$\begin{array}{c} \min{\left\|\alpha \right\|}_{1}, \end{array}$$

(6) $$\begin{array}{c} \underset{\alpha }{\min}\lambda {\left\|\alpha \right\|}_{1}+{\left\|FD_{l}\alpha -Fy\right\|}_{2}^{2}. \end{array}$$

Formula (6) is the generalized Lagrangian multiplier algorithm of the equivalent formula (5). The first term is the sparsity measurement, the second term is the sparse representation error, and *λ* is the balance coefficient. This problem is essentially a linear regression of the sparsity coefficient *λ* under the *L*1-norm. There are various dictionary learning methods, such as *K*-SVD and OMP methods. This article uses Matlab package to solve the dictionary, multiplying the obtained sparse coefficient *α* and the high-resolution dictionary *D*_*h*_ to reconstruct the corresponding high-resolution image. The flowchart of image reconstruction algorithm under sparse representation is shown in Figure 3.

(7) $$\begin{array}{c} x=D_{h}\alpha . \end{array}$$

### 2.3. Proposed Loss Function of Joint Dictionary

This section may be divided by subheadings. It should provide a concise and precise description of the experimental results, their interpretation, and the experimental conclusions that can be drawn.

The single dictionary in the image field is mainly used for sparse representation of the image. Its training process is as follows: (1) calculate the feature space of the input image blocks set *X*=[*x*_1_, *x*_2_,…*x*_*a*_], *x*_*i*_ ∈ *R*^*n*^,  *i*=1,2,…, *a*; (2) find the conditions of the dictionary *D*_*n*×*k*_: each image feature block can be adaptively and sparsely represented by certain base combinations in the dictionary optimally. This requires that the representation error is small enough and the coefficients are sparse enough to be represented by formula (6), where the representation coefficients of the dictionary and the feature block are both pending items. The research on the training algorithm of a single dictionary is mainly an optimization algorithm that satisfies two conditions. Usually this is an iterative process that includes two optimization processes. The two processes in the iteration include two optimizations of dictionary and coefficient.

Training the joint dictionary requires the use of high-resolution image block sets and low-resolution image block sets. On one hand, the feature space of the image block that needs to be extracted includes both high-resolution image block feature space *X* and low-resolution image block feature space *Y*. The image features extracted here must meet the condition that if *X* is regarded as a mapping to *Y*, then the extracted feature satisfies invariance or the mapping function. This condition is the focus of the construction of the mapping relationship between *X* and *Y* and has an important impact on the final reimage effect; on the other hand, it is mainly about sparse representation, that is, to obtain the sparse representation coefficient *α*_*l*_ of the low-resolution image block and pass the mapping relationship or the invariance relationship to obtain the representation coefficient *α*_*h*_ of the high-resolution image block, and then it reconstructs the high-resolution image.

The image blocks corresponding to the two feature spaces of image block are cascaded to form a new image feature block space. Assume that the training image block satisfies *P*={*Y*^*l*^, *X*^*h*^}, and *X*^*h*^={*x*_1_, *x*_2_,…, *x*_*n*_}, *Y*^*l*^={*y*_1_, *y*_2_,…, *y*_*n*_} represent the features extracted from the high- and low-resolution image blocks. *M* and *N* are the dimensions of the low-dimensional image feature block and the high-dimensional image feature block, respectively. The objective function of the loss function optimization-based joint dictionary fusion learning for superresolution MR imaging is described as

(8) $$\begin{array}{c} \underset{\left\{D_{h},D_{l},\alpha \right\}}{\min}\left\|X_{c}-D_{c}\alpha \right\|+\lambda \left(\frac{1}{N}+\frac{1}{M}\right){\left\|\alpha \right\|}_{1}, \end{array}$$

where $X_{c}=\left[\begin{array}{c} \left(1/\sqrt{N}\right)X^{h}\\ \left(1/\sqrt{M}\right)Y^{l} \end{array}\right]$, $D_{c}=\left[\begin{array}{c} \left(1/\sqrt{N}\right)D_{h}\\ \left(1/\sqrt{M}\right)D_{l} \end{array}\right]$, $D_{h}=\underset{\left\{D_{h},\alpha \right\}}{\arg\min}{\left\|X^{h}-D_{l}\alpha \right\|}_{2}^{2}+\lambda {\left\|\alpha \right\|}_{1}$, *D*_*l*_=argmin_{*D*_*l*_, *α*}_‖*Y*^*l*^ − *D*_*l*_*α*‖_2_^2^+*λ*‖*α*‖_1_. The image blocks and feature blocks have the same sparse representation coefficient with respect to the corresponding dictionary and then loss function for the dictionary training of the two image feature spaces. The dictionary pairs meet the requirements of being trained with the training image block *P*={*Y*^*l*^, *X*^*h*^}, and *X*^*h*^={*x*_1_, *x*_2_,…, *x*_*n*_}, *Y*^*l*^={*y*_1_, *y*_2_,…, *y*_*n*_}. In the training of joint dictionary loss function, the cascading error is used, which is the sum of the reconstruction error of low-resolution image blocks and the reconstruction error of high-resolution image blocks.

## 3. Proposed Joint Dictionary with Loss Function Optimization

According to (8), the features and problems of the joint dictionary are as follows: The training object is the set of two image blocks *P*={*Y*^*l*^, *X*^*h*^} after feature extraction; feature selection is very important. The gradient features of the first- and second-order gradients (image texture and edge information) are used here, and it is assumed that the corresponding feature blocks in the two feature spaces have the same sparse representation coefficients. The reconstruction error of low-resolution image feature dictionary is not guaranteed, nor is the reconstruction error of high-resolution image feature dictionary. Instead, the sum of error after cascading is solved by weighting. This paper proposes an optimization algorithm of the joint dictionary loss function, aiming at solving the problems of the joint dictionary. Its optimization idea is shown in Figure 4.

The mapping relationship between the two feature spaces is *y*_*i*_=Γ(*x*_*i*_), and Γ(•) can be linear or both nonlinear and unknown. For any image block {*y*_*i*_, *x*_*i*_}, the ideal dictionary pair {*D*_*y*_, *D*_*x*_} satisfies the following equations:

(9) $$\begin{array}{c} C_{i}=\underset{\alpha_{i}}{\arg\min}{\left\|y_{i}-D_{y}\alpha_{i}\right\|}_{2}^{2}+\lambda {\left\|\alpha \right\|}_{1},\;\forall i=1,\ldots ,N,\\ C_{i}=\underset{\alpha_{i}}{\arg\min}{\left\|x_{i}-D_{x}\alpha_{i}\right\|}_{2}^{2},\;\forall i=1,\ldots ,N, \end{array}$$

{*x*_*i*_}_*i*=1_^*N*^ represents the training sample in space *X*, {*y*_*i*_}_*i*=1_^*N*^ is the training sample in space *Y*, and {*c*_*i*_}_*i*=1_^*N*^ is the sparse representation coefficient. For a given input image *y*, the process of obtaining a high-resolution image block *x* is as follows: (1) obtain the sparse coefficient; (2) estimate *x*=*D*_*x*_*c* so that the reconstructed image block's error is minimized, namely:

(10) $$\begin{array}{c} L\left(D_{x},D_{y},x,y\right)=\left(\frac{1}{2}\right){\left\|D_{x}c-x\right\|}_{2}^{2}. \end{array}$$

Then the optimization formula of the optimized dictionary pair {*D*_*x*_^*∗*^, *D*_*y*_^*∗*^} is

(11) $$\begin{array}{c} \underset{D_{x,}D_{y}}{\min}\frac{1}{N}\overset{N}{\underset{i=1}{\sum }}L\left(D_{x},D_{y},x_{i,}y_{i}\right),s.t.\left\{\begin{array}{c} z_{i}=\underset{\alpha }{\arg\min}{\left\|y_{i}-D_{y}\alpha \right\|}_{2}^{2}+\lambda {\left\|\alpha \right\|}_{1},\;i=1,\ldots ,N,\\ {\left\|D_{x}\left(:,k\right)\right\|}_{2}\leq 1,\left\|D_{y}\left(:,k\right)\right\|\leq 1,\;k=1,\ldots ,K. \end{array}\right.. \end{array}$$

In order to ensure that the input image block *y* can be well represented by the dictionary *D*_*y*_, the reconstruction error function is added:

(12) $$\begin{array}{c} L=\left(\frac{1}{2}\right)\left[\gamma {\left\|D_{x}c_{i}-x_{i}\right\|}_{2}^{2}+\left(1-\gamma \right){\left\|D_{y}c_{i}-y_{i}\right\|}_{2}^{2}\right],0<\gamma \leq 1. \end{array}$$

Formula (12) is a nonlinear and nonconvex function, and it is optimized using an iterative optimization method.

The first step: Fix *D*_*y*_; then the optimization formula becomes

(13) $$\begin{array}{c} \underset{D_{x}}{\min}\overset{N}{\underset{i=1}{\sum }}\frac{1}{2}{\left\|D_{x}c_{i}-x_{i}\right\|}_{2}^{2},\\ \text{s.t.}\left\{\begin{array}{c} c_{i}=\underset{\alpha }{\arg\min}{\left\|y_{i}-D_{y}\alpha \right\|}_{2}^{2}+\lambda {\left\|\alpha \right\|}_{1},\;i=1,\ldots ,N\\ {\left\|D_{x}\left(:,k\right)\right\|}_{2}\leq 1,\;k=1,\ldots ,K. \end{array}\right. \end{array}$$

This is a quadratic programming problem with quadratic constraints, which can be solved by the conjugate gradient descent method.

The second step: Fix *D*_*x*_ and optimize *D*_*y*_. The minimization formula (15) is a two-layer optimization problem. The upper optimization is based on the variable *z*_*i*_, which is a low-level *ℓ*^1^ minimization problem. The gradient descent method is used to find a suitable gradient descent direction and then apply the chain derivative rule of differentiation.

(14) $$\begin{array}{c} \frac{\partial L}{\partial D_{y}}=\frac{1}{2}\left\{\underset{j\in \Omega }{\sum }\frac{\partial \left[\gamma R_{x}+\left(1-\gamma \right)R_{y}\right]}{\partial c_{i}}\frac{dc_{i}}{dD_{y}}+\left(1-\gamma \right)\frac{\partial R_{y}}{\partial D_{y}}\right\},џ\left\{\begin{array}{c} R_{x}={\left\|D_{x}c-x\right\|}_{2}^{2}\\ R_{y}={\left\|D_{y}c-y\right\|}_{2}^{2} \end{array}\right.. \end{array}$$

*c*_*j*_ is the *j* th element of *c*, and Ω is the index set of *j*. Suppose that $\tilde{c}$ is the index in {*c*_*j*_}_*j*∈Ω_ corresponding to Ω. $\tilde{D_{x}}$ and $\tilde{D_{y}}$ are subsets of *D*_*x*_ and *D*_*y*_; then:

(15) $$\begin{array}{c} \frac{\partial R_{x}}{\partial \tilde{c}}=2{\tilde{D}}_{x}^{T}\left(D_{x}c-x\right),\frac{\partial R_{y}}{\partial \tilde{c}}=2{\tilde{D}}_{y}^{T}\left(D_{y}c-y\right),\frac{\partial R_{y}}{\partial D_{y}}=2\left(D_{y}c-y\right)c^{T}. \end{array}$$

For the derivative $d\tilde{c}/dD_{y}$, use the following algorithm to calculate the derivative:

(16) $$\begin{array}{c} \frac{\partial {\left\|y-D_{y}c\right\|}_{2}^{2}}{\partial c_{j}}+\lambda \text{sign}\left(c_{j}\right)=0,\text{ for }j\in \Lambda =\left\{j|c_{j}\neq 0\right\}. \end{array}$$

Let Ω={*j|*|*c*_*j*_| > 0^+^}; therefore:

(17) $$\begin{array}{c} \frac{\partial {\left\|y-\tilde{D_{y}}\tilde{c}\right\|}_{2}^{2}}{\partial c_{j}}+\lambda \text{sign}\left(c_{j}\right)=0,\text{for j}\in \Omega . \end{array}$$

Equivalently find $\tilde{D_{y}^{T}}{\tilde{D}}_{y}\tilde{c}-{\tilde{D}}_{y}^{T}y+\lambda \text{sign}\left(\tilde{c}\right)=0$, where $\tilde{c}$ is a continuous function of *D*_*y*_. Use implicit derivation:

(18) $$\begin{array}{c} \frac{\partial \left\{{\tilde{D}}_{y}^{T}{\tilde{D}}_{y}\tilde{c}-{\tilde{D}}_{y}^{T}y\right\}}{\partial \tilde{D_{y}}}=\frac{\partial \left\{-\lambda *\text{sign}\left(\tilde{c}\right)\right\}}{\partial \tilde{D_{y}}},\\ \Rightarrow \frac{\partial {\tilde{D}}_{y}^{T}{\tilde{D}}_{y}}{\partial \tilde{D_{y}}}\tilde{z}+{\tilde{D}}_{y}^{T}{\tilde{D}}_{y}\frac{\partial \tilde{z}}{\partial \tilde{D_{y}}}-\frac{\partial {\tilde{D}}_{y}^{T}\tilde{c}}{\partial \tilde{D_{y}}}=0. \end{array}$$

Therefore:

(19) $$\begin{array}{c} \frac{\partial \tilde{c}}{\partial \tilde{D_{y}}}={\left({\tilde{D}}_{y}^{T}\tilde{D_{y}}\right)}^{-1}\left(\frac{\partial {\tilde{D}}_{y}^{T}y}{\partial \tilde{D_{y}}}-\frac{\partial {\tilde{D}}_{y}^{T}{\tilde{D}}_{y}}{\partial \tilde{D_{y}}}\tilde{c}\right). \end{array}$$

Here, the solution is required to be unique and $\left({\tilde{D}}_{y}^{T}{\tilde{D}}_{y}\right)$ exists. In order to solve formula, the gradient element *dz*/*dD*_*y*_=0 is maintained.

The joint dictionary pair training process based on loss function optimization used in this paper is shown in Figure 5.

## 4. Results and Analysis of the Experiment

### 4.1. Data and Settings of the Experiment

 This paper proposes an optimization algorithm of the joint dictionary loss function, aiming at solving the problems of the joint dictionary. The frame optimization idea is shown in Figure 4. The mapping relationship between the two feature spaces is, and can be linear or both nonlinear and unknown.

The data set in this paper mainly uses *T*1-weighted images (*T*1WI) and *T*2-weighted images (*T*2WI) from MR image sequences, which are derived from the open source data set. Different tissues have different signal intensity and image gray level in *T*1WI and *T*2WI. Small sample spatial data sets are formed due to differences in magnetic resonance equipment, magnetic field intensity, and imaging location. Among them, the small sample spatial data set includes neck, ankle transverse section, ankle longitudinal section, neck, head, major artery, carotid artery, knee, foot, and other human body parts, and the total number of samples from each part is about 70 on average. An example of the dataset is shown in Figure 6.

This paper adopts the superresolution reconstruction algorithm framework of MR image and uses the optimized joint dictionary loss function for training. 10 images were selected from the open source MR dataset as the sample for dictionary training. The initial parameters are set as follows: dictionary size is 512, balance parameter *λ* is 0.1, block size is 5 × 5, overlap block is 4, and the number of sample blocks is 150,000. The dictionary generated by training is shown in Figure 7.

### 4.2. Results and Analysis of the Experiment

The traditional dictionary training method requires a large number of training samples to ensure the validity of the training dictionary block. The more the training samples, the richer the prior knowledge, and the trained dictionary can make the reconstructed image closer to the actual image. However, sample abundance does not guarantee the validity of training samples. Poor quality samples can not only improve the quality of image reconstruction, but also reduce the effect of superresolution reconstruction. Therefore, this paper adopts the method in quality screening to screen the quality of training samples to ensure the complexity of training sample data. In the experiment, in order to compare the effect of image reconstruction, the original MR image data was taken as high-resolution image data, and the corresponding low-resolution image was obtained by double-cubic downsampling. Two training data sets and test data sets with different superresolution scales are obtained, which are ×2 and ×4, respectively. PSNR and SSIM were used to evaluate the reconstruction quality of MR images by different superresolution algorithms.

Firstly, the influence of various parameters on the performance of dictionary learning is analyzed, and the optimal combination of parameters is found. The following group of experiments show that a set of dictionaries are generated with the change of image block size, and the image effect is reconstructed under the same test image with different block conditions. Other parameters remain unchanged, and the variable parameter is the size of image block. The image block of the dictionary is consistent with that of the test image. When the superresolution ratio is 1 : 2, eight high-resolution dictionaries with blocks from 3 × 3 to 10 × 10 are generated in the experiment, and three of them are taken as shown in Figure 8. You can see that as the image block size increases, the dictionary block becomes more complex. The PSNR/SSIM values obtained are shown in Table 1.

PSNR and SSIM values of superresolution reconstruction generated by training dictionaries of different image blocks corresponding to test samples are shown in Table 1. The data is plotted using dictionary blocks and PSNR/SSIM as coordinates, as shown in Figures9 and 10. The abscissa of the data points in Figures 9 and 10 only represents the segmentation of the dictionary and the image. For example, the abscissa indicates that the segmentation of the dictionary is 5 × 5 and so on. As can be seen from the figure, when the size of overlapping blocks remains unchanged, increasing the block size will reduce PSNR value and SSIM value. In other words, the bigger the block, the better. If the block size is larger, the number of dictionary blocks represented by dictionary blocks will increase for an image feature block, which will increase the reconstruction error. It can be concluded from the figure that the optimal dictionary block value is 5 × 5.

At superresolution ratio 1:4 experiment generated block is 5 × 5 to 9 of 13 × 13 high-resolution dictionary, the three high-resolution dictionary is shown in Figure 11. It can be seen in the figure with the increase of chunking dictionary more and more complex, but it was too big block lead to too much when calculating the dictionary block singular matrix, which makes the dictionary piece of information loss, block the less effective dictionary block, the greater the results is. This results in a decrease in PSNR and SSIM.

The data in Table 2 are the corresponding PSNR values and SSIM values generated by superresolution reconstruction of test samples with different block training dictionaries. In order to distinguish the influence of block on reconstruction more intuitively, a graph with abscissa of image block and ordinate of PSNR/SSIM is drawn, as shown in Figure 11.

The abscissa in the figure only represents the segmentation of the image. It can be seen from the figure that the optimal PSNR/SSIM value corresponds to 10 × 10 image blocks. It can be seen that the feature of image blocks being too small indicates insufficiency, while the feature of image blocks being too large indicates limitations of the algorithm itself. By comparing the results of superresolution ratios 1 : 4 and 1 : 2, they have their own optimal blocks. The image blocks of superresolution ratio 1 : 4 are basically two times as large as the image blocks of superresolution ratio 1 : 2. This is because the local information of the image required by the 4-fold superresolution becomes larger, and the image blocks naturally become larger accordingly.

In the former two experiments, the fixed overlap block is 4, but in the overlap block experiment, the larger the overlap, the better. The experiment did not consider the best situation of the overlap block. Next, we use the corresponding maximum situation of different overlap blocks to see whether the best block changes. The experimental parameters are the same as above experiment. The changing parameters are only block size and overlapped block. For example, the block size is *n* × *n*. The value of overlap block is *n* − 1. Under the condition of superresolution ratio of 1 : 2, the experimental results are shown in Table 3. The data in the table represent the PSNR/SSIM value of superresolution reconstruction of each test sample under the corresponding blocks and overlapping blocks. The data are drawn as Figure 12 for more intuitive comparison.

In Figure 12 abscissa of data points indicate only the dictionary blocks. For example, abscissa 5 indicates that the dictionary blocks are 5 × 5, and so on. As can be seen from the figure, it is still better to use the 5 × 5 dictionary for reconstruction, too small blocks have insufficient features, too large blocks need more pixels to be calculated, and the increase of dictionary representation blocks caused by larger feature blocks will increase errors and affect PSNR/SSIM values. In this experiment, the maximum overlap block is used to achieve the best reconstruction condition for each component block. It can be seen that the optimal block value is still 5 × 5.

When the superresolution ratio is 1 : 4, the experimental results are shown in Table 4. The obtained data were plotted with block size as abscissa and PSNR/SSIM as ordinate, as shown in Figure 13. As can be seen from the figure, when the superresolution ratio is 1 : 4, the superresolution reconstruction effect of the dictionary divided into 10 × 10 training blocks is the best. As can be seen from the above experiments, the block size has a maximum value and is related to the superresolution ratio. The larger the superresolution ratio is, the larger the required block will be, and the change of overlapping blocks will not change the result of the optimal block. For MR images, the optimal block with the superresolution ratio of 1 : 2 is 5 × 5 and the optimal block with the superresolution ratio of 1 : 4 is 10 × 10.

Using the same parameters, the variable parameter is the sampling number of image sample blocks, which can be overlapped to extract data. The superresolution ratio is 1 : 2. The experimental results are shown in Table 5. The data in the table are sampled from image blocks and the trained dictionaries are taken as abscissa and PSNR/SSIM as ordinate to draw an image, as shown in Figure 14.

It can be seen from Figure 14 that 10000 pieces of the following samples quantity is too little, because in the algorithm they do not conform to the requirements of the sample piece, MR images have a lot of black or dark area is larger, the gray level change is not big, and at zero or near zero all samples will be removed, which makes the actual participation in computing block greatly reduced. Therefore, as a training sample block, there are not enough features to reduce the value of PSNR/SSIM during reconstruction. On the contrary, the great increase of the number of blocks does not bring great changes to PSNR/SSIM, and there is no maximum value, showing fluctuations. All the training sample blocks are involved in the dictionary training. Too many blocks will increase the training time and have no positive significance for the generation of high-definition dictionaries. Therefore, it can be seen from the figure that 150,000 sample blocks should be selected. The following is an experimental verification of the superresolution ratio of 1 : 4. The data in Table 6 were sampled from image blocks with different numbers of trained dictionaries as abscissa and PSNR/SSIM as ordinate to draw an image, as shown in Figure 15.

As can be seen from the figure, superresolution ratio 1 : 4 and superresolution ratio 1 : 2 have the same conclusion in block selection, while superresolution ratio 1 : 4 cannot train the dictionary when the number of blocks is 1000, so it has higher requirements on the number of dictionaries. In consideration of reducing the dictionary training time, it is appropriate to choose the number of 150,000 blocks.

Several parameters affecting the superresolution effect are analyzed, and the optimal parameters of the superresolution MR image are obtained, as shown in Table 7.

Finally, we have the comprehensive comparison, and Table 8 shows the reconstruction effects of different superresolution methods, including bicubic interpolation, nearest neighbor, joint dictionary learning, and our superresolution method based on joint dictionary loss function optimization, where the values highlighted in bold are the best under the corresponding image quality evaluation indexes. It can be seen from Table 8 that the joint dictionary loss function optimization method we proposed is optimal in both the neck and ankle reconstruction results.

Compared with bicubic interpolation, nearest neighbor, and joint dictionary, the PSNR of the proposed method is 2.61 dB, 5.69 dB, and 0.45 dB higher on ×2 superfractal scale on average. SSIM increased by 0.0317, 0.0688, and 0.0059 on average. Compared with the original combined dictionary, the maximum improvement of PSNR value and SSIM value after optimization is about 1 dB and 0.0088, respectively. The average improvement of PSNR of reconstruction quality on ×4 superscale was 1.30 dB, 4.84 dB, and 0.25 dB, respectively. The average SSIM increases by 0.0321, 0.0944, and 0.0057. Compared with the original combined dictionary, the maximum improvement of PSNR value and SSIM value after optimization is about 0.85 dB and 0.0065, respectively. The results of image reconstruction show that the proposed superresolution method based on error loss function optimization is superior to other algorithms.

### 4.3. Discussion

As experimental results, the original image features are directly used to carry out the superresolution algorithm, and the computational efficiency will be low due to the huge amount of data. Joint dictionary fusion learning has widely used imaging, feature extraction, and classification. The high-resolution and low-resolution dictionaries are trained and ensure that all the features of image blocks exist in the dictionaries. The dictionary is redundant; that is, the different image blocks are represented with several representations. We optimize the loss function of dictionary learning with the joint high- and low-resolution dictionary block pair and increase the high-resolution reconstruction error. Experiments show that, compared with algorithms such as bicubic interpolation, nearest neighbor, and original dictionary learning, the algorithm in this paper has a better superdivision reconstruction performance. With the future applications, our proposed method in our paper is superior to the original superresolution image reconstruction with double sparse representation dictionary learning. The advantage including the proposed algorithm applies the objective function of the loss function optimization-based joint dictionary fusion learning, which improves the performance of image reconstruction from the low resolution to high resolution. The disadvantage lies in that the novel loss function will increase a little complexity of the time consuming compared with the original optimization. Some results are shown in Table 9. Because the computing consuming of the superresolution algorithm is not high, the computing is little for the application. The proposed dictionary learning-based MR superresolution is feasible and effective for the applications. The method only uses the low-resolution and high-resolution images for the different parts of the body, and it does not need all high-resolution and low-resolution images from the same person. In the practical applications, it is necessary to train the dictionary with the training samples including the MR contrast and body part. Our method does not need the training to be separate for different parts of the body, and they only train one time for acquisition parameters including different TE, TRs, etc.

## 5. Conclusion

This paper proposes a superresolution algorithm of MR image based on joint dictionary loss function optimization. In order to solve the problem that the joint dictionary loss function applies cascading error and does not guarantee the reconstruction error of the high-resolution image dictionary, the algorithm constructs a new loss function, ensuring that while the sparse coefficients are sparse enough, in the iterative training process, the high- and low-resolution dictionaries are trained separately to reduce the error generated by the joint high- and low-resolution dictionary block and increase the high-resolution reconstruction error, thus ensuring that the learned high-resolution dictionary can well reconstruct the MR image. In order to verify the effectiveness of the algorithm, a comparative experiment was carried out with a variety of superresolution algorithms, and a quantitative analysis was carried out based on the experimental results. The results show that the proposed algorithm has a better reconstruction effect in MR image superresolution and maintains the best effect in large-scale superresolution at the same time. The proposed method in this paper further improves the application performance of the joint dictionary superresolution method on MR images and also provides an experimental framework and method for subsequent MR image superresolution.

## Figures and Tables

**Figure 1:** MR image superresolution architecture based on joint dictionary training.

**Figure 2:** Sparse representation of MR image blocks.

**Figure 3:** The flow of image superresolution algorithm under sparse representation.

**Figure 4:** Dictionary loss function optimization.

**Figure 5:** Joint dictionary pair training based on loss function optimization.

**Figure 6:** MR test images.

**Figure 7:** Training dictionary after loss function optimization.

**Figure 8:** High-resolution dictionary blocks (superresolution 1 : 2). (a) The dictionary is 3 × 3. (b) The dictionary is 6 × 6. (c) The dictionary is 10 × 10.

**Figure 9:** Superresolution PSNR/SSIM values of dictionary images constructed with different blocks (superresolution ratio 1 : 2). (a) The curve of PSNR value changing with dictionary block. (b) The curve of SSIM value changing with dictionary block.

**Figure 10:** High-resolution dictionary blocks (superresolution 1 : 4). (a) The dictionary is 5 × 5. (b) The dictionary is 9 × 9. (c) The dictionary is 13 × 13.

**Figure 11:** Superresolution PSNR/SSIM values of dictionary images constructed with different blocks (superresolution ratio 1 : 4). (a) The curve of PSNR value changing with dictionary block. (b) The curve of SSIM value changing with dictionary block.

**Figure 12:** Comparison of superresolution PSNR/SSIM for different blocks of a dictionary (superresolution ratio 1 : 2). (a) The curve of PSNR value. (b) The curve of SSIM value.

**Figure 13:** Comparison of superresolution PSNR/SSIM for different blocks of a dictionary (superresolution ratio 1 : 4). (a) The curve of PSNR value. (b) The curve of SSIM value.

**Figure 14:** PSNR/SSIM value corresponding to the training dictionary using different number of samples (superresolution ratio 1 : 2). (a) The curve of PSNR value changing with the number of samples. (b) The curve of SSIM value changing with the number of samples.

**Figure 15:** PSNR/SSIM value corresponding to the training dictionary using different number of samples (superresolution ratio 1 : 4). (a) The curve of PSNR value changing with the number of samples. (b) The curve of SSIM value changing with the number of samples.

**Table 1:** The PSNR/SSIM values using different block constructed dictionaries (superresolution 1 : 2).

Dictionary block size	Sample set 1	Sample set 2	Sample set 3	Sample set 4	Sample set 5
5 × 5	32.24/0.9407	28.87/0.8996	32.04/0.9302	30.59/0.9145	30.34/0.9208
6 × 6	32.30/0.9412	28.87/0.8984	32.06/0.9309	30.53/0.9060	30.31/0.9084
7 × 7	31.99/0.9328	28.75/0.8875	31.95/0.9251	30.32/0.9025	30.14/0.9003
8 × 8	31.62/0.9297	28.44/0.8716	31.65/0.9195	30.09/0.8894	29.89/0.8936
9 × 9	31.20/0.9158	28.21/0.8658	31.33/0.9102	29.80/0.8721	29.52/0.8835
10 × 10	30.92/0.9021	27.95/0.8513	31.18/0.9031	29.60/0.8684	29.27/0.8748

**Table 2:** The PSNR/SSIM values under different dictionary blocks (superresolution ratio 1 : 4).

Dictionary block size	Sample set 1	Sample set 2	Sample set 3	Sample set 4	Sample set 5
5 × 5	29.82/0.8755	25.34/0.7913	29.16/0.8758	27.09/0.8172	27.54/0.8201
6 × 6	30.00/0.8778	25.49/0.7948	29.38/0.8782	27.22/0.8315	27.72/0.8285
7 × 7	30.30/0.8813	25.61/0.7996	29.49/0.8799	27.18/0.8243	27.91/0.8366
8 × 8	30.40/0.8857	25.71/0.8107	29.72/0.8823	27.23/0.8366	28.02/0.8434
9 × 9	30.43/0.8902	25.69/0.8238	29.78/0.8904	27.27/0.8430	28.05/0.8541
10 × 10	30.75/0.9008	25.75/0.8323	29.94/0.8987	27.32/0.8503	28.11/0.8635
11 × 11	30.67/0.8912	25.77/0.8285	29.90/0.8922	27.22/0.8354	28.12/0.8634
12 × 12	30.53/0.8905	25.71/0.8274	29.82/0.8913	27.19/0.8255	27.93/0.8413
13 × 13	30.31/0.8821	25.60/0.8002	29.64/0.8810	27.08/0.8141	27.78/0.8224

**Table 3:** Comparison of superresolution PSNR/SSIM for different block and overlap block training dictionaries (superresolution ratio 1 : 2).

Block size	Overlapped block	Sample set 1	Sample set 2	Sample set 3	Sample set 4	Sample set 5
3 × 3	2	31.30/0.9154	28.21/0.8639	31.22/0.8966	30.26/0.9013	29.70/0.8944
4 × 4	3	31.96/0.9273	28.70/0.8834	31.73/0.9143	30.54/0.9087	30.19/0.9123
5 × 5	4	32.24/0.9407	28.87/0.8996	32.03/0.9302	30.59/0.9145	30.34/0.9208
6 × 6	5	32.29/0.9411	28.90/0.9001	32.07/0.9297	30.55/0.9102	30.32/0.9175
7 × 7	6	32.11/0.9328	28.83/0.8926	32.03/0.9274	30.40/0.9056	30.26/0.9122
8 × 8	7	31.90/0.9240	28.71/0.8854	31.93/0.9203	30.26/0.9048	30.08/0.9068
9 × 9	8	31.71/0.9188	28.60/0.8738	31.80/0.9185	30.10/0.9003	29.93/0.9002
10 × 10	9	31.43/0.9201	28.42/0.8687	31.65/0.9033	29.95/0.8875	29.70/0.8917

**Table 4:** Comparison of superresolution PSNR for different block and overlap block training dictionaries (superresolution ratio 1 : 4).

Block size	Overlapped block	Sample set 1	Sample set 2	Sample set 3	Sample set 4	Sample set 5
3 × 3	2	29.22/0.8619	25.05/0.7746	28.78/0.8607	26.91/0.8014	27.11/0.8273
4 × 4	3	29.45/0.8677	25.16/0.7832	28.93/0.8704	26.97/0.8085	27.26/0.8344
5 × 5	4	29.82/0.8755	25.34/0.7913	29.16/0.8758	27.09/0.8172	27.54/0.8401
6 × 6	5	30.19/0.8824	25.57/0.7988	29.43/0.8812	27.26/0.8200	27.81/0.8503
7 × 7	6	30.63/0.8875	25.72/0.8104	29.68/0.8875	27.30/0.8276	28.06/0.8556
8 × 8	7	30.80/0.8908	25.88/0.8233	29.96/0.8908	27.35/0.8302	28.25/0.8623
9 × 9	8	30.92/0.8994	25.94/0.8399	30.03/0.8966	27.43/0.8483	28.30/0.8701
10 × 10	9	31.11/0.9109	25.96/0.8487	30.15/0.9043	27.44/0.8514	28.31/0.8722
11 × 11	10	30.91/0.9025	25.91/0.8410	30.09/0.9002	27.32/0.8311	28.22/0.8614
12 × 12	11	30.87/0.8902	25.90/0.8315	30.05/0.8954	27.30/0.8292	28.17/0.8600
13 × 13	12	30.63/0.8843	25.76/0.8184	29.88/0.8871	27.19/0.8145	27.98/0.8496

**Table 5:** The PSNR/SSIM value corresponding to the number of sample blocks of different sampling images (superresolution ratio 1 : 2).

Number of sample image blocks	Sample set 1	Sample set 2	Sample set 3	Sample set 4	Sample set 5
1000	31.98/0.8945	28.64/0.8735	31.74/0.9101	30.45/0.8997	30.10/0.9043
5000	32.15/0.9076	28.79/0.8804	31.94/0.9189	30.52/0.9021	30.23/0.9067
10000	32.20/0.9207	28.81/0.8861	31.96/0.9184	30.56/0.9076	30.28/0.9112
50000	32.29/0.9412	28.84/0.8922	31.99/0.9245	30.57/0.9132	30.31/0.9183
100000	32.24/0.9407	28.87/0.9011	32.03/0.9302	30.59/0.9145	30.34/0.9208
150000	32.31/0.9413	28.91/0.9003	32.04/0.9301	30.60/0.9166	30.37/0.9207
200000	32.26/0.9409	28.84/0.8937	32.04/0.9308	30.58/0.9152	30.35/0.9211
500000	32.32/0.9415	28.86/0.8986	32.01/0.9255	30.61/0.9105	30.35/0.9200

**Table 6:** The PSNR/SSIM value corresponding to the number of sample blocks of different sampling images (superresolution ratio 1 : 4).

Number of sample image blocks	Sample set 1	Sample set 2	Sample set 3	Sample set 4	Sample set 5
1000	—	—	—	—	—
5000	29.78/0.8625	25.29/0.7820	29.11/0.8679	27.04/0.8026	27.43/0.8247
10000	29.75/0.8632	25.30/0.7838	29.15/0.8712	27.09/0.8134	27.48/0.8296
50000	29.77/0.8714	25.35/0.7916	29.16/0.8745	27.11/0.8196	27.53/0.8377
100000	29.82/0.8755	25.34/0.7913	29.16/0.8758	27.09/0.8172	27.54/0.8401
150000	29.84/0.8761	25.38/0.7924	29.18/0.8832	27.08/0.8195	27.54/0.8412
200000	29.81/0.8759	25.36/0.7908	29.17/0.8807	27.09/0.8187	27.51/0.8407
500000	29.85/0.8764	25.39/0.7923	29.16/0.8776	27.10/0.8201	27.53/0.8411

**Table 7:** Optimal parameters of MR image superresolution.

Superresolution ratio	Equilibrium parameters	Overlapped block	Dictionary block size	Number of sampling blocks
1 : 2	0.1	4	5 × 5	150000
1 : 4	0.1	9	10 × 10	150000

**Table 8:** Comparison of the quality of several superresolution reconstructed images.

Image	The multiple of image superresolution	Bicubic interpolation	Nearest neighbor image block	Joint dictionary	Dictionary optimization algorithm
Neck1	2	37.84/0.9473	33.19/0.9002	40.29/0.9751	41.24/0.9839
	4	30.84/0.8856	26.92/0.8027	31.95/0.9042	31.98/0.9102

Neck2	2	34.30/0.9166	30.57/0.8695	37.78/0.9503	38.09/0.9584
	4	27.74/0.8211	25.70/0.7834	29.10/0.8497	29.95/0.8562

Neck3	2	35.50/0.9004	31.31/0.8712	36.68/0.9179	36.95/0.9203
	4	28.80/0.8329	26.28/0.7998	30.05/0.8712	30.14/0.8744

Ankle1	2	31.31/0.8834	30.03/0.8587	34.57/0.9199	35.07/0.9257
	4	26.72/0.8003	22.07/0.7105	27.56/0.8262	27.74/0.8310

Ankle2	2	30.52/0.8781	28.92/0.8398	32.48/0.9087	32.55/0.9132
	4	25.50/0.7858	22.40/0.7416	26.31/0.8200	26.31/0.8211

Ankle3	2	33.26/0.9072	30.21/0.8708	33.89/0.9163	34.48/0.9214
	4	29.06/0.8587	24.05/0.7729	30.02/0.8711	30.35/0.8842

**Table 9:** Comparison of time consuming of several superresolution reconstructed images (ms).

Image	The multiple of image superresolution	Bicubic interpolation	Nearest neighbor image block	Joint dictionary	Dictionary optimization algorithm
Neck1	2	35.7	43.1	65.9	**75.5**
	4	42.4	49.7	69.4	**74.8**

Neck2	2	36.3	44.2	66.2	**74.3**
	4	41.3	49.4	69.2	**75.2**

## Data Availability

The authors have not used specific data from other sources for the simulations of the results. The popular MR datasets in this paper are of free download from the website https://www.mr-tip.com/serv1.php?type=db. The proposed algorithm is implemented in python.
